RETRACTED

# Detection and Genotyping of *Francisella tularensis* in Animal Hosts and Vectors from Six Different Natural Landscape Areas, Gansu Province, China

**DOI:** 10.1155/2021/6820864

**Published:** 2021-12-18

**Authors:** Fang Zhang, Xiaoheng Wang, Guowei Yu, Jiangli Gao, Hongmei Niu, Jin Zhao

**Affiliations:** ^1^Faculty of Medicine, Northwest Minzu University, Lanzhou 730030, China; ^2^Key Laboratory of Environmental Ecology and Population Health in Northwest Minority Areas, Northwest Minzu University, Lanzhou 730030, China

## Abstract

**Objective:**

Tularemia, also known as hare fever, is caused by the bacterium *Francisella tularensis* (*F. tularensis*) transmitted through diseased wild animals, blood sucking insects, or contaminated water or food, which is distributed worldwide. The purpose of this study was to investigate *F. tularensis* infection in animal hosts and vectors from six different natural landscape areas in Gansu Province and to identify the genotypes of the detected *F. tularensis*.

**Methods:**

Rodents were captured by snap traps, and ticks were collected by dragging a cloth over the vegetation or from domestic animals. After species identification, DNA was isolated from the captured animals and detected by nested PCR assays targeting the *F. tularensis* fopA gene. The positive samples were further amplified to discriminate the species, and another two short-sequence tandem repeat regions (SSTR) were amplified to identify their genotypes. All positive fragments were sequenced and analyzed by ClustalX (5.0) and DNAClub software.

**Results:**

A total of 407 rodents of 12 species were captured, among which six rodent species were positive for *F. tularensis*, with an overall prevalence of 3.93%. The geographical difference in infection rate was statistically significant. At the SSTR9 locus, there were 7 genotypes among positive rodent samples. A total of 1864 ticks were tested for evidence of tularemia by nested PCR assays, 69 of which were positive, with an average positive rate of 3.70% for *F. tularensis* in ticks. The positive rates were significantly different among different regions. Seven genotypes were identified at the SSTR9 locus, one of which seemed dominant in positive tick samples. All positive samples had the same genotype at the SSTR16 locus.

**Conclusion:**

There is natural infection of *F. tularensis* among animal vectors and hosts in Gansu Province, with diverse genotypes.

## 1. Introduction

Tularemia, or hare fever, is a natural focal disease caused by *Francisella tularensis* (*F. tularensis*) transmitted through diseased wild animals, blood sucking insects, or contaminated water or food, which is distributed worldwide [1, 2]. The hosts of tularemia in nature mainly include arthropods and mammals, such as ticks, hares, and rodents [3]. Tularemia is caused by gram-negative and facultative intracellular tularemia, and the organism is classified as a biological agent due to its extremely low infection dose and high mortality [4]. Two subspecies are responsible for the majority of tularemia cases, namely, *F. tularensis* subsp. *tularensis* (*Ftt*) and *F. tularensis subsp. holarctica* (*Fth*). The most virulent strains of Ftt may induce severe pneumonia, with a fatality rate of up to 30% [5].

RETRACTED

In China, *F. tularensis* was first reported in 1957 [6]. In 1959, Heilongjiang Province reported the first human infection with hare fever [7]. Subsequently, natural foci of tularemia were confirmed in Tibet, Xinjiang, and Gansu [8, 9]. Pathogenic bacteria were isolated from patients with hare fever, ticks, rabbits, and mice in the above areas. The latest outbreak occurred in 1986 at a food processing factory in Shandong Province, where 31 of 36 workers who slaughtered hares became ill [10]. Since then, there have been no more reported cases of natural “hare fever” or *F. tularensis* infection among animal hosts in China. At present, it is not clear whether the natural foci have disappeared or are at a standstill in the past or just because they were not reported. In addition, many of the epidemiological characteristics of the disease, such as infection of other hosts, changes of foci, and genotypic differences, remain unclear. In recent years, Polymerase Chain Reaction (PCR) technology has been widely used to detect host *F. tularensis* infection [11, 12]. However, molecular technology is extremely expensive and requires advanced laboratory facilities and technical expertise, limiting its application in resource-poor endemic diseases [13]. Conventional single-step PCR (CPCR), real-time quantitative PCR (qPCR), nested PCR (NPCR), and PCR-restriction fragment length polymorphism (PCR-RFLP) have been widely used in the detection of different gene sequences. Despite its popularity in disease diagnosis, PCR amplification has some inherent drawbacks, such as high DNA similarities between species, leading to primer mismatches, and low copy numbers of specific genes for pathogen identification [14]. NPCR is a modification of CPCR, using two sets of primers and two consecutive PCR reactions. NPCR was invented to increase the amplification efficacy in terms of detection limit and amplification specificity [15].

Previous studies have shown that *F. tularensis* exists in some areas of Gansu Province [16, 17]. This study is the first to conduct epidemiological investigations of animal hosts and vectors infected with tularemia in 6 different natural landscape areas. As the ecological environment in China is complex and diverse, the potential vectors and hosts of tularemia are diverse and widely distributed, with great regional differences. In addition, ticks of different species in different regions also have great differences in the incidence of tularemia. *F. tularensis* has 4 subspecies, which differ greatly in terms of epidemiological characteristics such as geographic distribution, animal hosts, virulence, and transmission routes. Short tandem repeat sequences are the result of strand-slippage during DNA replication and are widely found in prokaryotes and eukaryotes. The genotyping method based on sequence polymorphism has been successfully applied to many pathogens including *F. tularensis*, with encouraging results [18, 19]. Preliminary experiments with laboratory strains of *F. tularensis* have demonstrated through laboratory animals that the SSTR locus remained stable on plates after numerous passages. In this study, we used this method to select the two most commonly used gene regions and perform further genotyping analysis on the positive samples. The results showed that there were 9 different genotypes of *F. tularensis*, although all of them belonged to subspecies B.

RETRACTED

In this study, animal hosts and vectors of tularemia in six different natural landscape areas from Gansu Province were tested to *F. tularensis* and to determine the subspecies type of the agent using PCR technology, which contributes to a better understanding of the natural infection of tularemia in Gansu Province as well as the status and the natural foci of the disease. In addition, we used short sequence tandem repeat (SSTR) polymorphism to genotype the positive specimens and combined with epidemiological data to determine the relationship between genotypes and geographic distribution, animal host, transmission route, etc., laying a foundation for the molecular epidemiological study of tularemia in Gansu Province.

## 2. Object and Method

### 2.1. On-Site Epidemiological Investigation and Specimen Collection

The investigation was conducted in the following six natural landscape areas in Gansu Province: Longxi area, Longdong area, Longnan area, Gannan area, Qilianshan area, and Hexi corridor area. Tick specimens were acquired using the flagging method [20] or collected from the surface of animals. Tick species from different habitats are collected and kept in a suitable environment for laboratory processing. Rodents were captured with baited snap traps [21]; that is, the snap traps were placed in the evening and retrieved in the early morning of the next day to trap rodents in different habitats. After species and sex (only male rates were collected) were identified, sterile anatomical specimens were collected on site, and the spleen tissue was collected and stored at -20°C for later use. The sample collection time was from April 2019 to July 2019.

RETRACTED

### 2.2. DNA Sample Preparation

After the identification of rodents, about 3 mm^3^ (about 500 mg) of spleen tissue was aseptically cut and added with Trizol (Gibco), which was placed in a sterile grinder and fully ground into an eppendorf tube. After removing the RNA by centrifugation, DNA precipitation was obtained after two washings (0.1 mol/L sodium citrate 10% ethanol solution). Then, it was suspended in 75% alcohol and let stand for 10-20 min, followed by centrifugation at 2000 × g for 5 min at 2-8°C.The DNA particles were then dissolved overnight in 8 mmol/L NaOH solution at 4°C. Finally, the extracted DNA was dissolved in TE (0.01 mol/L, pH 8.0) and stored at -20°C for use. The concentration and purity of the DNA were measured with an ultraviolet spectrophotometer (Vilber Lourmat, France). For tick specimens, after the identification of tick species, they were soaked in 75% alcohol for 20 minutes, blotted dry with sterile filter paper, and rinsed with normal saline 3 times. After absorbing the moisture on the tick's body surface with sterile filter paper, the ticks were placed in PE tubes and added with 50-200 *μ*L DNA extraction buffer (10 mM Tris, pH 8.0, 2 mM EDTA, 0.1% SDS, 500 *μ*g of protease K/ml) to grind thoroughly with a sterilized pipette tip. After that, they were incubated at 56°C for 2 hours, boiled in boiling water for 10 minutes, and stored at -20°C for later use.

### 2.3. PCR Amplification

Five pairs of primers were used to detect the samples (Table 1), among which the universal set of primers FNA8L/FNA2L (outer side) and FNA7L/FNA1L (inner side) amplified the *fopA* gene of tularemia [3]. The C6/C8 pairs are species-specific primers, which can be used to distinguish the two subspecies of *F. tularensis* A and B through the different lengths of the amplified fragments. For the specimens with positive *fopA* gene amplification, two pairs of primers, 9F/9R and 16F/16R, were used to amplify the SSTR9 and SSTR16 loci of the *F. tularensis* gene for genotyping analysis [5]. The primers used, which can be found in Table 1, were synthesized by (Beijing) Tiangen Company. All amplifications were performed on the ABI2700 PCR machine (Applied Biosystems, USA).

### 2.4. Product Detection, Recovery, and Purification

The amplification results were detected by 1.5% agarose gel electrophoresis, and positive PCR products were recovered by DNA fragment recovery kit (Qiagen, UK). All operations are carried out in strict accordance with the instructions.

RETRACTED

### 2.5. Nucleic Acid Sequence Determination and Analysis

The recovered fragments were sent to Invitrogen for sequencing. The sequencing results were analyzed and compared using ClustalX (5.0), DNAClub, and MEGA (4.0). Other known fragment sequences were from NCBI GenBank (website: http://www.ncbi.nlm.nih.gov).

### 2.6. Statistical Analysis

The *χ*2 test and the Fisher exact probability method were used to compare the differences in infection rates among different regions, different animal hosts, and vectors, and the SPSS (23.0) software was used for statistical processing.

## 3. Results

### 3.1. Animal Host Infection

A total of 407 rodents were captured (Table 2), including 12 species such as *Apodemus* and *Cricetulus*. Among them, 16 specimens of 6 rodent species were amplified by nested PCR to produce a 409 bp fragment (Figure 1), and the overall positive rate of *F. tularensis* was 3.93%. Among the six positive rodent species, *Meriones unguiculatus* had the highest positive rate, reaching 25%, followed by *Eutamias sibiricus*, 20%. Although there were differences in the positive rates among different species, there was no significant difference. The positive rate was different in 6 different natural landscape areas (*χ*2 = 15.06, *P* < 0.01), with the highest positive rate of 11.54% in Qilian mountain area. It was 7.85% in Longdong area and 3.57% in Gannan area. No positive specimens were detected in other areas. There was no difference in the positive rate of rodent species in various regions.

### 3.2. Infection of Animal Vectors

More than 3,000 ticks were caught in 6 different natural landscape areas, while only 1864 adult ticks and non-blood-sucking ticks were used for detection. There were 8 tick species including *Dermacentor nuttalli*, *Dermacentor Dagestan*, *Hyalophthalmia qinghaiensis*, *Dermacentor savanna*, *Ixodes persulcatus*, *Haemaphysalis qinghaiensis*, *Haemaphysalis longicornis*, and Persian ticks. Among them, 69 ticks from 6 tick species and 4 natural landscape areas tested positive, with a total positive rate of 3.7% (Table 3).

The highest positive rate of *F. tularensis* was found in *Dermacentor* ticks, which was 9.59%, followed by *Haemaphysalis longicornis* 6.38%, *Haemaphysalis qinghaiens* 6.10%, *Dermacentor nuttalli* 6.04%, *Dermacentor Dagestan* 5.71%, and *Ixodes persulcatus* 1.74%. The species of *Hyalopia asiatica* and *Persian sharp* tick were not detected. The positive rate was significantly different among different tick species (*χ*2 = 33.04, *P* < 0.05). A comparison of the positive rates of 6 different natural landscape areas found that there was a difference (*χ*2 = 20.51, *P* < 0.05). The positive rate in Longdong area was the highest, which was 10.27%.

RETRACTED

### 3.3. Subspecies Identification of Positive Specimens

Subspecies-specific primers (C6/C8) were used for further subspecies identification of the amplified positive specimens (Figure 2). The target bands (220 bp fragment) were amplified from 69 tick specimens and 16 mouse specimens, and the nucleic acid sequences were sequenced and retrieved (GenBank, website: http://www.ncbi.nlm.nih.gov). It was found to be 100% homologous to the sequence AF247690.2 of *F. tularensis subsp. B* in the database.

### 3.4. Analysis of SSTR9 and SSTR16 Sites in Positive Specimens

The sequence at the SSTR16 locus was identical in the specimens (Figure 3(a)), with a fragment size of 361 bp and a repetitive sequence of AAGATATTTGTAGAAA (copy number: 2). There were 9 different copy numbers at the SSTR9 locus, which were 7, 8, 9, 10, 14, 15, 16, 18, and 21, indicating that there were 9 different genotypes at this locus, expressed as copy numbers. The distribution of genotypes in each specimen is shown in Table 4.

The copy number of the repetitive sequence at the SSTR9 locus of rodents ranged from 8 to 21 (Table 4), and the size of the amplified fragment ranged from 314 to 396 bp (Figure 3(b)). The copy numbers at the SSTR9 locus of specimens in the same area were not exactly the same. There were multiple copies of specimens in Longdong area, including 8, 10, 14, 15, and 16; 3 specimens in Qilian area had 8, 15, 18, and 3 copy number. The specimens in Gannan area were 18 and 21 forms. Tick specimens had 7 genotypes at the SSTR9 locus, of which the two genotypes with copy numbers 9 and 15 accounted for the majority: 42 out of the 69 specimens were of these two types. The distribution of other genotypes is shown in Table 4.

### 3.5. Cluster Analysis of Positive Specimens Based on SSTR9 Region Sequence

Using the MEGA (4.0) software, cluster analysis was performed based on the SSTR9 locus sequence of positive specimens (Figure 4). The results showed that the positive specimens mainly clustered into three large groups, namely, ticks, rodents, and mixed groups; specimens from various regions did not show strict regional characteristics, and there was a clear crossover of genotypes at this locus.

## 4. Discussion

Gansu Province is located at the intersection of Qinghai Tibet Plateau, Mengxin plateau, and Loess Plateau in China. The whole territory is divided into 6 natural landscape areas (types), namely, low mountains, hills, dry grassland, and semidesert area of Loess Plateau in western Gansu; Gully steppe and semidesert area of Loess Plateau in Eastern Gansu; mountain forest and grassland area in South Gansu; Gannan plateau, canyon alpine meadow grassland, grassland, forest, and forest grassland area; Qilian Mountain, alpine grassland, and forest grassland area; and Hexi Corridor semidesert, desert grassland, and Gobi desert area. In this area, the neighboring sections move to each other, the topography is diverse, the climate change is obvious, the ecological environment is diverse, and the vegetation and various animal species are various and abundant. There are multiple animal hosts and geographic landscapes suitable for the survival and prevalence of multiple pathogens. In principle, the incidence of tularemia is similar to that of *borreliosis*, in which the incidence of pathogens in tick nymphs is negatively correlated with altitude [22].

RETRACTED

The results confirmed the presence of *F. tularensis* in Gansu Province. In previously identified foci, bacterial DNA was detected in both the ticks and rodents, which confirmed to a certain extent that the past foci still existed. There have been no case reports in recent years, but that does not mean the foci has disappeared or subsided. Of the six natural landscape areas detected, only the Hexi Corridor area has not detected positive specimens, but it cannot be ruled out that there is no tularemia bacteria in this area. In the future, we can expand the survey sampling sites and collect more samples for further exploration. In the study, the Tianshui Maiji Mountain Scenic Area was selected as the survey sampling site in the eastern Gansu area. The pathogens were detected in wild rodents and ticks, which to a certain extent, indicated that the Maiji Mountain Scenic Area may be a natural focus of tularemia. It confirmed that the disease will pose a potential threat to tourists in the scenic area, which warrants special attention from the local health department. Among several other natural landscape areas, Qilian, Gannan, and Longnan areas have been identified as natural foci of tularemia in previous studies. So, it is not surprising that pathogens were detected in the animal hosts and vectors in this study, as the foci of past outbreaks have not disappeared, and we should continue to pay attention to them in the future. At the same time, health education for local residents should be strengthened, and personal protection should be taken when entering the foci of the foci, which is essential for disease prevention.

At present, about 250 species of animals have been found to be the vectors and hosts of *F. tularensis*, among which rodents and blood-sucking arthropods are the most important natural hosts and vectors. In this study, a total of 12 different species of rodents and 8 species of ticks were captured in Gansu Province. These animal hosts and vectors are all dominant and common species in the region. Among them, 6 rodent species and 6 tick species tested positive. However, due to the limited number of specimens collected from some species and the fact that only one test has been conducted, the results may be biased. In addition, since we have not yet conducted any transmission dynamics experiment, it is impossible to determine which species are currently available through this study. Moreover, future continuous monitoring and related experiments should be carried out to explain which rodent and which tick species and why they are the dominant host and vector species of *F. tularensis* in Gansu Province.

RETRACTED

This fully illustrates the diversity and complexity of the genotypes of *F. tularensis* in Gansu Province. Based on the SSTR9 locus, the cluster analysis of *F. tularensis* showed that the specimens were mainly divided into three major groups, tick colonies, rodent colonies, and mixed groups. *F. tularensis* from different specimen sources showed certain specificity, especially in ubiquitous genotypes in tick specimens, suggesting that there may be species-specific genotypes in *F. tularensis*, which is consistent with the results of Goethert [20]. It is necessary to systematically carry out relevant research on pathogens.

The COVID-19 epidemic is another wake-up call for biosecurity. At the critical moment, the Central Committee decided to “integrate biological safety into the national security system in order to protect people's health, safeguard national security and maintain the country's long period of stability and stability.” *F. tularensis* is highly infectious, pathogenic, and easily transmitted. Many Western countries such as the United States have listed it as a bioterrorist pathogen along with anthrax, plague, and smallpox. Although the pathogen is widespread in northern China [3–6, 12, 13], it has not attracted enough attention. The incubation period of tularemia is usually 3 to 5 days but can be extended to 14 days. Systemic symptoms include fever, malaise, chills, and headache. However, there are six typical presentations of tularemia in humans, including glandular ulcer, glandular ulcer, pneumonia ulcer, oropharyngeal ulcer, ocular gland ulcer, and systemic ulcer. In most cases, the location and route of infection determine the clinical form of the disease [21]. Unfortunately, no vaccine against tularemia is available or approved for use in humans at present. Under the increasingly severe form of antiterrorism, countries where natural conditions in favor of tick-borne infection in humans and animals need to formulate disease management strategies and establish control schemes for tick-borne diseases. It is urgent to conduct detailed and systematic research on pathogens so that the nature of the disease can be determined and the source of pathogens can be traced when the disease occurs. Meanwhile, long-term monitoring of the foci should be carried out to understand the changing situation and take active measures to prevent problems before they happen. On the other hand, the possible impact of climate change, urbanization, and industrial and agricultural pollution on infectious diseases should be considered. It is recommended that regional disease control plans be implemented to fight against infectious diseases with the concept of One Health [23].

RETRACTED

In conclusion, this study was the first to explore *F. tularensis* infection in animal hosts and vectors from six different natural landscape areas in Gansu Province, and it was found that *F. tularensis* infection existed in 5 different natural landscape areas with high genetic diversity. There are some limitations. Animals of different genders may present different genotypes, so more detailed species types are needed to comprehensively study the genotyping of *F. tularensis* in animal hosts and vectors from different areas.

## Figures and Tables

**Figure 1:** Prevalence of *F. tularensis* in rodents. 1-4 and 7-12: test negative specimens; 5: test positive specimens; 6: 100 bp marker; 13: negative control.

**Figure 2:** Amplification results in C6/C8 region. 1-8: test positive specimens.

**Figure 3:** Amplification results in SSTR9 and SSTR16 regions: (a) SSTR16; (b) SSTR9. 1-10: different genotypes of *F. tularensis*.

**Figure 4:** The cluster analysis based on SSTR9 region.

**Table 1:** Primers and PCR condition used in the study.

Primers	(5′-3′) sequence	Cycle parameters	Length (bp)
FNA8L	CGAGGAGTCTCAATGTACTAAGGTTTGCCC	95°C 3 min →95°C 15 s, 55°C 15 s, 72°C 30 s, 35 cycles→72°C 10 min	900
FNA2L	CACCATTATCCTGGATATTACCAGTGTCAT		
FNA7L	CTTGAGTCTTATGTTTCGGCATGTGAATAG		409
FNA1L	CCAACTAATTGGTTGTACTGTACAGCGAAG		
C6	TCCGGTTGGATAGGTGGTGGATT	94°C 5 min →94°C 30 s, 64°C 30 s, 72°C 30 s, 30 cycles→72°C 10 min	220/250A
C8	GCGCGGATAAATTTAAATTC		
9F	GTTTTCACGCTTGTCTCCTATCA	94°C 5 min →94°C 30 s, 62°C 30 s,72°C 30 s, 30 cycles→72°C 10 min	200~400
9R	CAAAAGCAACAGCAAAATTCACAAA		
16F	GTTGGCGAACCTAAAATAATAGC	94°C 5 min →94°C 30 s, 60°C 30 s,72°C 30 s, 30 cycles→72°C 10 min	300~500
16R	CAGCTCGAACTCCGTCATC		

A: the amplified fragment length of subspecies A was 250 bp and that of subspecies B was 220 bp.

**Table 2:** Prevalence of *F. tularensis* in rodents.

Rodent species	Number of positive/detected						
	Longdong	Longxi	Hexi	Qilian	Gannan	Longnan	Total
*Apodemus peninsulae*	9/43	0/12	0/5	—	—	—	9/60
*Apodemus agrarius*	0/24	0/12	—	—	2/36	0/7	2/79
*Cricetulus barabensis*	0/23	0/37	0/15	—	—		0/75
*Cricetulus migratorius*	—	—	—	1/4	0/13		1/17
*Tscherskia triton*	1/5	—	—	—	—		1/5
*Myodes rufocanus*	—	—	0/5	—	—	—	0/5
*Rottus losea*	—	—	—	—	—	0/5	0/5
*Rattus norvegicus*	0/17		0/10	0/7	02	0/5	0/41
*Mus musculus*	0/15	0/17	0/24	0/12	0/2	—	0/70
*Allactaga sibirica*	0/10	0/11	0/15	—	—	—	0/36
*Meriones unguiculatus*	—	—	—	1/4	—		1/4
*Eutamias sibiricus*	1/3	—	—	1/4	—	0/3	2/10
Total	11/140	0/99	0/66	3/26	2/56	0/20	16/407

RETRACTED

**Table 3:** Prevalence of *F. tularensis* in ticks.

Tick species	Number of positive/detected						
	Longdong	Longxi	Hexi	Qilian	Gannan	Longnan	Total
*Hyalomma asiaticum*	—	—	0/237	0/110	—	—	0/347
*Argas persicus*	—	—	0/124	0/95	—	—	0/219
*Dermacentor nuttalli*	15/102	4/54	0/98	—	14/233	8/192	41/679
*Dermacentor silvarum*	5/44	—	—	—	2/29	—	7/73
*Haemaphysalis longicornis*	—	9/141	—	—	—	—	9/141
*Dermacentor Dagestan*	2/35	—	—	—	—	—	2/35
*Haemaphysalis qinghaiensis*	5/82	—	—	—	—	—	5/82
*Ixodes persulcatus*	—	—	—	—	2/110	3/178	5/288
Total	27/263	13/195	0/459	0/205	18/372	11/370	69/1864

**Table 4:** Distribution of genotypes from samples.

Genotypes	Rodent samples	Tick samples
7		PD-1
8	SD-1, SQ-1	PX-8, PG-(13-18)
9		PD-(3-11), PD-(21-27), PX-(1-6), PG-(1-5)
10	SD-8	PL-(1-5)
14	SD-2, SD-7	PL-(6-11)
15	SQ-2, SD-5, SD-9	PG-7, PG-8, PD-(12-20), PX-(7-13)
16	SD-3, SD-4, SD-6, SD-10, SD-11	PG-(9-12)
18	SQ-3, SG-1	PD-2
21	SG-2	

S: rodent specimens; P: tick specimens; D: Longdong; X: Longxi; H: Hexi; Q: Qilian; G: Gannan; L: Longnan; 1 (2,...,69): positive sample No.

## Data Availability

The labeled datasets used to support the findings of this study are available from the corresponding author upon request.
